The article "Chimeric ZHHH neuroglobin acts as a cell membrane‐penetrating inducer of neurite outgrowth" was published in 2017. Journal: FEBS Open Bio.

# Chimeric ZHHH neuroglobin acts as a cell membrane‐penetrating inducer of neurite outgrowth

**DOI:** 10.1002/2211-5463.12271

**Published:** 2017-08-14

**Authors:** Nozomu Takahashi, Wataru Onozuka, Seiji Watanabe, Keisuke Wakasugi

**Affiliations:** ^1^ Department of Life Sciences Graduate School of Arts and Sciences The University of Tokyo Japan; ^2^ Present address: Department of Neuroscience and Pathobiology Research Institute of Environmental Medicine Nagoya University Nagoya Aichi Japan

**Keywords:** cell membrane‐penetrating protein, neurite outgrowth, neuroglobin, rat pheochromocytoma PC12 cell line

## Abstract

Neuroglobin (Ngb) is a heme protein expressed in the vertebrate brain. We previously engineered a chimeric Ngb protein, in which module M1 of human Ngb is replaced by that of zebrafish Ngb, and showed that the chimeric ZHHH Ngb has a cell membrane‐penetrating activity similar to that of zebrafish Ngb and also rescues cells from death caused by hypoxia/reoxygenation as does human Ngb. Recently, it was reported that overexpression of mammalian Ngb in neuronal cells induces neurite outgrowth. In this study, we performed neurite outgrowth assays of chimeric Ngb using rat pheochromocytoma PC12 cells. Addition of chimeric Ngb, but not human or zebrafish Ngb, exogenously to the cell medium induces neurite outgrowth. On the other hand, the K7A/K9Q chimeric Ngb double mutant, which cannot translocate into cells, did not induce neurite outgrowth, suggesting that the cell membrane‐penetrating activity of the chimeric Ngb is crucial for its neurite outgrowth‐promoting activity. We also prepared several site‐directed chimeric Ngb mutants and demonstrated that residues crucial for neurite outgrowth‐inducing activity of the chimeric Ngb are not exactly the same as those for its neuroprotective activity.

**Abbreviations**
DMEM: Dulbecco's modified Eagle's medium
GDI: guanine nucleotide dissociation inhibitor
Gα_i/o_: α‐subunit of heterotrimeric G_i/o_ protein
Ngb: neuroglobin
NGF: nerve growth factor
WT: wild‐type

Neuroglobin (Ngb) is an oxygen‐binding heme protein that has a classical globin fold and is expressed in the vertebrate nervous system 1, 2, 3, 4, 5, 6, 7, 8. Mammalian Ngb proteins are involved in the neuronal response to hypoxia and ischemia and protect neurons from hypoxic–ischemic insults 9, 10, 11, 12, 13. Expression of mammalian Ngb was reported to increase in response to neuronal hypoxia *in vitro* and to focal cerebral ischemia *in vivo* 9, 14. Mammalian Ngb was also reported to protect the brain from experimentally induced stroke *in vivo* 14, 15.

We previously demonstrated that human Ngb binds to flotillin‐1, a lipid raft microdomain‐associated protein, and exists in lipid rafts only during oxidative stress and that translocation of human Ngb to lipid rafts under oxidative stress conditions is crucial for neuroprotection by Ngb 13, 16. Moreover, we found that human Ngb binds exclusively to the GDP‐bound form of the α‐subunits of heterotrimeric G_i/o_ proteins (Gα_i/o_), which are present in lipid rafts and inhibit adenylate cyclase activity, thereby acting as guanine nucleotide dissociation inhibitor (GDI) for Gα_i/o_ and inhibiting the reduction in intracellular cAMP concentration to protect against cell death 13, 17, 18, 19, 20, 21, 22.

Although Ngb was originally identified in mammalian species, it is also present in nonmammalian vertebrates 23, 24. Fish Ngb proteins are also hexacoordinated globins with similar oxygen‐binding kinetics 24. We showed that zebrafish Ngb does not exhibit GDI activity and cannot rescue cell death 10, 11, 19, 25. Moreover, by using FITC‐labeled Ngb proteins, we found that zebrafish but not human Ngb can translocate into cells 11. Using site‐directed mutagenesis, we showed that K7A/K9Q and K21Q/K23Q double mutants of zebrafish Ngb are unable to translocate 25, 26, suggesting that Lys7, Lys9, Lys21, and Lys23 of zebrafish Ngb play important roles in zebrafish Ngb protein transduction. In addition, we demonstrated that cellular uptake of zebrafish Ngb is dependent on negatively charged cell surface glycosaminoglycan 27. A probable mechanism of zebrafish Ngb protein transduction is electrostatic interaction of the protein with glycosaminoglycan on the plasma membrane, followed by penetration into cells by macropinocytosis, and subsequent release from endosome to cytoplasm 28.

The genes encoding human and zebrafish Ngb each comprise four exons interrupted by three introns. Exons 1, 2, 3, and 4 correspond to compact protein structural ‘modules’, termed M1, M2, M3, and M4, respectively 18, 19, 23, 24, 29. We previously engineered a chimeric Ngb protein, in which module M1 of human Ngb is replaced by that of zebrafish Ngb, as shown in Fig. 1, and showed that the chimeric ZHHH Ngb acts as a GDI for Gα_i/o_ and rescues PC12 cells from death caused by hypoxia/reoxygenation, as does human Ngb 10, 19. Moreover, we demonstrated that chimeric ZHHH Ngb can translocate into cells and protect them from cell death 11.

**Figure 1:** Schematic representation of the human, zebrafish, and chimeric ZHHH Ngb proteins used in this study. The genes of human and zebrafish Ngb comprise four exons interrupted by three introns; exons 1, 2, 3, and 4 encode compact protein structural ‘modules’, termed M1, M2, M3, and M4, respectively. Module M1 of human Ngb was replaced by that of zebrafish Ngb to produce the chimeric ZHHH Ngb protein.

Recently, it was reported that overexpression of human or mouse Ngb protein in neuronal cells induces neurite outgrowth 30, 31. Therefore, in this study, we first examined whether chimeric ZHHH Ngb functions as a novel cell membrane‐penetrating inducer of neurite outgrowth by using rat pheochromocytoma PC12 cells, as PC12 cells have been widely used as a model for investigating neuronal differentiation and neurite outgrowth 32, 33, 34. Neurite‐specific genes are induced in PC12 cells and neurite outgrowth occurs after stimulation with nerve growth factor (NGF) 33, 34. After evaluating the neurite outgrowth‐inducing activity of the chimeric ZHHH Ngb, we prepared several site‐directed mutants of the chimeric ZHHH Ngb to clarify which residues of chimeric ZHHH Ngb are crucial for its neurite outgrowth activity.

## Materials and methods

### Preparation of Ngb proteins

Plasmids expressing human Ngb, zebrafish Ngb, and chimeric ZHHH Ngb, in which module M1 of human Ngb was replaced by that of zebrafish Ngb, were prepared as described previously 17, 19. A QuikChange™ site‐directed mutagenesis system (Stratagene, La Jolla, CA, USA) was used to introduce substitutions at specific sites. The constructs were confirmed by DNA sequencing (FASMAC Co., Ltd., DNA sequencing services, Atsugi, Japan). Overexpression of each Ngb protein was induced in *Escherichia coli* strain BL21 (DE3) after treatment with isopropyl‐β‐d‐thiogalactopyranoside, and each Ngb protein was purified as described previously 17, 19. In brief, soluble cell extracts were loaded onto DEAE Sepharose anion‐exchange columns equilibrated with buffer A (20 mm Tris/HCl, pH 8.0). Ngb proteins were eluted from the columns with buffer A containing 75 mm NaCl, and further purified by passage through Sephacryl S‐200 HR gel filtration columns. Purified Ngb was dialyzed overnight against phosphate‐buffered saline (PBS). Endotoxin was removed from the protein solutions by phase separation using Triton X‐114 (Sigma‐Aldrich, St. Louis, MO, USA) 35, 36. Trace amounts of Triton X‐114 were removed by passage through Sephadex G‐25 gel (GE Healthcare Biosciences, Piscataway, NJ, USA) equilibrated with PBS.

### Cell culture

A rat pheochromocytoma PC12 cell line (RCB0009) was obtained from the RIKEN Cell Bank (Ibaraki, Japan). PC12 cells were maintained in culture in Dulbecco's modified Eagle's medium (DMEM) containing 4.5 g·L^−1^ glucose, 10% (v/v) FBS, 10% (v/v) heat‐inactivated horse serum, 100 U·mL^−1^ penicillin, 100 μg·mL^−1^ streptomycin, and 2 mm glutamine (all from Invitrogen, Carlsbad, CA, USA) in a humidified atmosphere containing 5% CO_2_ at 37 °C. The medium was changed twice weekly, and the cultures were split 1 : 8 once every week.

### Neurite outgrowth assay

Mouse NGF 2.5S (Grade II) was purchased from Alomone Labs Ltd. (Jerusalem, Israel). PC12 cells were plated on 35‐mm, glass‐bottomed, poly‐d‐lysine‐coated (Sigma‐Aldrich) dishes (Iwaki; Asahi Techno Glass, Tokyo, Japan) or poly‐d‐lysine‐coated 96‐well tissue culture plates (Corning, Corning, NY, USA) at a density of 2.0 × 10^4^ cells·mL^−1^ in DMEM containing 4.5 g·L^−1^ glucose, 10% (v/v) FBS, 10% (v/v) heat‐inactivated horse serum, and 2 mm glutamine for 24 h. Each Ngb (10 μm) was added exogenously to the cell medium, or PBS or NGF (100 ng·mL^−1^) was added as a negative or positive control, respectively. The cells were incubated at 37 °C for 48 h under normoxia (95% air/5% CO_2_). The living PC12 cells were observed with differential interference contrast microscopy (Nikon C2 plus; Nikon Instruments, Tokyo, Japan) or phase contrast microscopy (Olympus IX71; Olympus, Tokyo, Japan). Cells with at least one neurite longer than 10 μm were defined as neurite‐bearing cells. We determined the percentage of neurite‐bearing cells relative to the total number of cells counted. Approximately 300 cells were counted in three random fields in each well.

For the 5‐day incubation, PC12 cells were plated on 35‐mm, glass‐bottomed, poly‐d‐lysine‐coated (Sigma‐Aldrich) dishes (Iwaki; Asahi Techno Glass) or poly‐d‐lysine‐coated 96‐well tissue culture plates (Corning) at a density of 5.0 × 10^3^ cells·mL^−1^ in DMEM containing 4.5 g·L^−1^ glucose, 10% (v/v) FBS, 10% (v/v) heat‐inactivated horse serum, and 2 mm glutamine for 24 h. Each Ngb (10 μm) was added exogenously to the cell medium, or PBS or NGF (100 ng·mL^−1^) was added as a negative or positive control, respectively. The PC12 cells were incubated at 37 °C for 5 days under normoxia (95% air/5% CO_2_). From the third day of incubation, half of the medium containing NGF (100 ng·mL^−1^) or Ngb (10 μm) was refreshed every day. After a total of 5 days, the living PC12 cells were observed with differential interference contrast or phase contrast microscopy. The cells that possessed at least one neurite more than one cell body diameter in length were defined as cells with long processes. We determined the percentage of cells with long processes relative to the total number of cells counted. Approximately 200 cells were counted in three random fields in each well.

### FITC labeling of Ngb proteins

Ngb was conjugated to FITC (Dojindo, Kumamoto, Japan) according to the instructions of a Fluoreporter® FITC protein labeling kit (Molecular Probes, Eugene, OR, USA). FITC‐labeled Ngb was purified using G25 gel chromatography to eliminate free FITC. Electronic absorption spectra of Ngb proteins were recorded with a UV‐visible spectrophotometer (UV‐2450; Shimadzu, Kyoto, Japan). The concentrations of Ngb protein and FITC dye in each purified FITC‐labeled Ngb protein were calculated on the basis of their absorbance at the Soret peak and 494 nm, respectively. The molar ratio of dye to protein in each purified FITC‐labeled Ngb protein was determined to be 0.9–1.3 FITC dye molecules per molecule of protein.

### Observation of protein translocation into cells with fluorescence microscopy

PC12 cells were seeded at 2 × 10^4^ cells·mL^−1^ in 35‐mm, glass‐bottomed, poly‐d‐lysine‐coated (Sigma‐Aldrich) dishes (Iwaki; Asahi Techno Glass) and incubated for 24 h. FITC‐labeled Ngb (3 μm) was then added to cells that had been washed in DMEM without serum. Fresh DMEM without serum was added and the cells were incubated at 37 °C for 1 h; FBS and FM4‐64 (Molecular Probes), a general fluorescent marker of endocytosis, were added to final concentrations of 2% and 1 μm, respectively. The cells were incubated under normoxia at 37 °C for 24 h. PC12 cells were washed with cold PBS twice, and the living, unfixed cells were directly observed with Nikon C2 plus confocal microscope (Nikon Instruments).

### Treatment of cells with Ngb protein and hydrogen peroxide

PC12 cells were plated on poly‐d‐lysine‐coated 96‐well tissue culture plates (Corning) at a density of 1.0 × 10^5^ cells·mL^−1^ in DMEM containing 4.5 g·L^−1^ glucose, 10% (v/v) FBS, 10% (v/v) heat‐inactivated horse serum, and 2 mm glutamine for 24 h. Each Ngb (10 μm) was added to cells that had been washed in DMEM without serum. Fresh DMEM without serum was added, and the cells were incubated at 37 °C for 1 h; FBS was then added to a final concentration of 2%. The cells were incubated at 37 °C for 24 h. The medium was then changed to fresh DMEM containing 4.5 g·L^−1^ glucose, 10% (v/v) FBS, 10% (v/v) heat‐inactivated horse serum, and 2 mm glutamine. The cells were then treated with 200 μm hydrogen peroxide for 24 h at 37 °C.

### Cell viability assay

Cell viability was measured with CellTiter 96® AQueous One Solution Cell Proliferation Assay Reagent (Promega, Madison, WI, USA), containing [3‐(4,5‐dimethylthiazol‐2‐yl)‐5‐(3‐carboxymethoxyphenyl)‐2‐(4‐sulfophenyl)‐2H‐tetrazolium, inner salt; MTS]. The cultured cells were incubated with the MTS reagent at 37 °C for 3 h in a humidified, 5% CO_2_ atmosphere. The amount of formed colored formazan was quantified by measuring absorbance at 490 nm with a Beckman Coulter DTX880 plate reader (Beckman Coulter, Fullerton, CA, USA).

## Results

### Neurite outgrowth‐promoting activity of chimeric ZHHH Ngb

We first tested the neurite outgrowth‐inducing activity of NGF in PC12 cells. Using differential interference contrast microscopy, undifferentiated PC12 cells were observed as round without neurites (Fig. 2A). PC12 cells responded to NGF by flattening of the cell body and subsequent extension of neurites (Fig. 2A). The percentages of neurite‐bearing cells with at least one neurite longer than 10 μm are summarized in Fig. 2B, which clearly shows that NGF significantly stimulates neurite outgrowth of PC12 cells.

**Figure 2:** Effects of NGF, WT chimeric ZHHH, human, zebrafish, and K7A/K9Q chimeric ZHHH Ngb proteins on neurite outgrowth of PC12 cells following 2 days of incubation. (A) Differential interference contrast images of PC12 cells incubated with PBS, NGF (100 ng·mL^−1^), or Ngb (10 μm). Scale bar, 10 μm. (B) Neurite outgrowth‐promoting activity of Ngb. The graphs show the percentages of neurite‐bearing cells with at least one neurite longer than 10 μm relative to the total number of cells counted. All data are expressed as means ± SEM from at least three independent experiments, each performed in triplicate. Data were analyzed by one‐way ANOVA followed by Tukey–Kramer *post hoc* tests. **P < 0.01 compared with PBS. (C) SDS/PAGE analysis of purified Ngb proteins. The samples were analyzed on 15.0% SDS/polyacrylamide gels and stained with Coomassie Brilliant Blue. The sizes in kilodaltons of molecular markers are indicated at the left. (D) Dose‐dependent effect of the WT chimeric ZHHH Ngb on neurite outgrowth in PC12 cells. All data are expressed as means ± SEM from three experiments. Data were analyzed by one‐way ANOVA followed by Tukey–Kramer *post hoc* tests. **P < 0.01 compared with PBS. ^##^ *P* < 0.01 compared with WT chimeric ZHHH Ngb.

We then prepared human, zebrafish, and chimeric ZHHH Ngb proteins and investigated their effects on neurite outgrowth of PC12 cells under differential interference contrast or phase contrast microscopy. The purity of Ngb proteins used in the experiments was confirmed by SDS/PAGE (Fig. 2C). The exposure of PC12 cells to chimeric ZHHH Ngb induced significant neurite outgrowth compared with PBS (Fig. 2A,B). Moreover, we also observed a dose–response effect of chimeric ZHHH Ngb on neurite outgrowth (Fig. 2D). In contrast, the exogenous addition of human or zebrafish Ngb to the cell medium did not induce neurite outgrowth (Fig. 2A,B).

### The neurite outgrowth‐promoting activity of chimeric ZHHH Ngb is dependent on its cell membrane‐penetrating activity

We prepared FITC‐labeled Ngb proteins and reconfirmed that both zebrafish and chimeric ZHHH Ngb, but not human Ngb, can penetrate the cell membrane of PC12 cells (Fig. 3) 11. Because the K7A/K9Q double mutant of zebrafish Ngb cannot penetrate the cells 25, 26, we next evaluated whether the FITC‐labeled K7A/K9Q chimeric ZHHH Ngb double mutant could penetrate the cell membrane of PC12 cells. As shown in Fig. 3, the K7A/K9Q double mutant did not translocate into cells. Moreover, the K7A/K9Q chimeric ZHHH Ngb double mutant did not induce significant morphological changes in PC12 cells (Fig. 2A,B). Taken together, these results indicate that translocation of chimeric ZHHH Ngb into PC12 cells is crucial for its neurite outgrowth‐promoting activity.

**Figure 3:** Transduction of FITC‐labeled WT and K7A/K9Q chimeric ZHHH, human, and zebrafish Ngb proteins into PC12 cells. About 3 μm of FITC‐labeled (green) Ngb protein was applied to PC12 cells in the presence of FM4‐64 (red), a fluorescent marker of endocytosis. The cells were then incubated for 24 h under normoxic conditions. The living, unfixed cells were observed directly by confocal fluorescence microscopy. Scale bar, 10 μm.

### Influence of the heme environmental structural change in chimeric ZHHH Ngb on its neurite outgrowth activity

The iron atom in the heme prosthetic group of Ngb normally exists in either the ferrous (Fe^2+^) or ferric (Fe^3+^) redox state. Both the ferric and ferrous bis‐His forms of Ngb are hexacoordinated to their endogenous protein ligands, namely proximal and distal His residues (Fig. 4), and oxygen can displace the distal His residue of ferrous Ngb to produce ferrous oxygen‐bound mono‐His Ngb 2.

**Figure 4:** Sequence alignment of human, zebrafish, and chimeric ZHHH Ngb proteins used in this study. Multiple sequence alignment was performed using the clustalw software (Kyoto University Bioinformatics Center, Kyoto, Japan) with manual adjustments. The positions of modules M1–M4 and α‐helices A–H (Protein Data Bank Code: 1OJ6) of human Ngb are shown above the sequences. Intron positions in human and zebrafish Ngb are indicated by arrows. Residues crucial for the GDI activity of human Ngb and the cell membrane‐penetrating activity of zebrafish Ngb are marked in blue and red, respectively. The proximal and distal His residues of human Ngb are marked in green. Numbers on the left and right of the sequences correspond to those at the beginning and end of the sequences, respectively. Gaps in the sequences are indicated by dashes. The residues corresponding to 53, 60, and 118 in human Ngb are highlighted in blue in chimeric ZHHH Ngb.

To investigate the effects of this structural change in chimeric ZHHH Ngb on its neurite outgrowth activity, we prepared an H67V chimeric ZHHH Ngb mutant, in which the distal His residue was substituted with Val, as a model of chimeric ZHHH Ngb that cannot form a bis‐His conformation. The purity of the Ngb protein used in the experiment was confirmed by SDS/PAGE (Fig. 5A). As shown in Fig. 5B,C, the H67V chimeric ZHHH Ngb still induced neurite outgrowth similar to wild‐type (WT) chimeric Ngb, suggesting that the heme environmental structural changes in chimeric ZHHH Ngb are not crucial for its neurite outgrowth activity.

**Figure 5:** Effects of WT, H67V, E56Q, E63Q, and E121Q chimeric ZHHH Ngb proteins on neurite outgrowth of PC12 cells following 2 days of incubation. (A) SDS/PAGE analysis of purified Ngb proteins. The samples were analyzed on 15.0% SDS/polyacrylamide gels and stained with Coomassie Brilliant Blue. The sizes in kilodaltons of molecular markers are indicated at the left. (B) Differential interference contrast images of PC12 cells incubated for 2 days with PBS or Ngb (10 μm). Scale bar, 10 μm. (C) Neurite outgrowth‐promoting activity of Ngb (10 μm). The graph shows the percentage of neurite‐bearing cells with at least one neurite longer than 10 μm relative to the total number of cells counted. All data are expressed as means ± SEM from at least four independent experiments, each performed in triplicate. Data were analyzed by one‐way ANOVA followed by Tukey–Kramer *post hoc* tests. **P < 0.01 compared with PBS. ^##^ *P* < 0.01 compared with WT chimeric ZHHH Ngb.

Moreover, differential interference contrast microscopy (Fig. 6A) of PC12 cells after the 5‐day incubation revealed that the percentage of cells with a process longer than one cell diameter was increased in the presence of WT chimeric ZHHH Ngb compared with PBS (Fig. 6B). H67V chimeric ZHHH Ngb also significantly increased neurite outgrowth (Fig. 6A,B), suggesting that the mono‐His form of Ngb induces neurite outgrowth.

**Figure 6:** Effects of NGF, WT chimeric ZHHH Ngb, human Ngb, zebrafish Ngb, K7A/K9Q chimeric ZHHH Ngb double mutant, and H67V, E56Q, E63Q, or E121Q chimeric ZHHH Ngb single mutants on neurite outgrowth of PC12 cells after 5 days of incubation. (A) Differential interference contrast images of PC12 cells incubated with PBS, NGF (100 ng·mL^−1^), or Ngb (10 μm) for 5 days. Scale bar, 10 μm. (B) The percentage of cells with processes longer than their cell body after 5 days of incubation. All data are expressed as means ± SEM from three independent experiments, each performed in triplicate. Data were analyzed by one‐way ANOVA followed by Tukey–Kramer *post hoc* tests. *P < 0.05, **P < 0.01 compared with PBS. ^##^ *P* < 0.01 compared with WT chimeric ZHHH Ngb.

### Search for residues crucial for the neurite outgrowth activity of chimeric ZHHH Ngb

As shown in Figs 2A,B, and 3, zebrafish Ngb penetrated into cells but did not induce neurite outgrowth, suggesting that human Ngb possesses different residues than the zebrafish Ngb and that these are important for the neurite outgrowth activity of human Ngb. To examine this possibility, we aligned and compared the amino acid sequences of human, zebrafish, and chimeric ZHHH Ngb proteins (Fig. 4). We previously demonstrated that the Glu53, Glu60, and Glu118 residues of human Ngb are crucial for its GDI and neuroprotective activities 10, 11, 13, 19, 21, 22. To investigate whether the residues crucial for neurite outgrowth‐promoting activity of human Ngb are the same as those for its GDI activity, we prepared E56Q, E63Q, and E121Q chimeric ZHHH Ngb single mutants, in which the corresponding Glu53, Glu60, and Glu118 residues of human Ngb in chimeric ZHHH Ngb were each mutated to Gln. The purities of the resulting Ngb proteins were confirmed by SDS/PAGE (Fig. 5A). E56Q chimeric ZHHH Ngb induced neurite outgrowth similar to WT chimeric ZHHH Ngb (Fig. 5B,C), which is consistent with a previous report showing E53Q human Ngb induces neurite outgrowth similar to WT human Ngb 30. On the other hand, neither E63Q nor E121Q chimeric ZHHH Ngb stimulated neurite outgrowth (Fig. 5B,C). As shown in Fig. 6A,B, after 5 days of incubation, WT and E56Q chimeric ZHHH Ngb, but not E63Q and E121Q chimeric ZHHH Ngb, increased the percentage of PC12 cells with processes longer than their cell bodies, suggesting that the Glu63 and Glu121 residues of chimeric ZHHH Ngb are crucial for its neurite outgrowth‐inducing activity.

### Neuroprotective activities of chimeric ZHHH Ngb mutants

We previously revealed human H64V Ngb, which cannot form the bis‐His conformation, did not act as a GDI for Gα_i1_ and did not protect cells from oxidative stress 13. We also showed that human E53Q, E60Q, and E118Q Ngb, which lack GDI activity, did not protect cells against oxidative stress‐induced cell death, suggesting that Glu53, Glu60, and Glu118 of human Ngb are crucial for its neuroprotective activity 10, 13, 21, 22. Therefore, we next investigated the effects of the corresponding residues of chimeric ZHHH Ngb on its neuroprotective activity.

Neuroglobin protein was added exogenously to the cell medium of PC12 cells, and the protective effect of Ngb protein against hydrogen peroxide‐induced cell death was tested. Cell viability was measured by MTS assays and is shown in Fig. 7. The absorbance at 490 nm obtained by MTS assay is directly proportional to the number of living cells 22. As shown in Fig. 7, cell survival was enhanced by WT chimeric ZHHH Ngb. This result is consistent with our previous results 10, 11, 12, 22. Next, we tested whether H67V chimeric ZHHH Ngb, in which the corresponding His64 of human Ngb in chimeric ZHHH Ngb was mutated to Val, can protect cells against hydrogen peroxide‐induced cell death. As shown in Fig. 7, H67V chimeric ZHHH Ngb did not rescue cell death during oxidative stress. Therefore, we confirmed that oxidative stress‐induced structural change in chimeric ZHHH Ngb is crucial for its neuroprotective activity. Moreover, we examined the protective effect of E56Q, E63Q, and E121Q chimeric ZHHH Ngb single mutants, in which the corresponding Glu53, Glu60, and Glu118 residues of human Ngb in chimeric ZHHH Ngb were each mutated to Gln, against cell death. MTS assays showed that these chimeric ZHHH Ngb mutants did not protect PC12 cells against hydrogen peroxide‐induced cell death (Fig. 7). Thus, we demonstrated that Glu56, Glu63, and Glu121 of chimeric ZHHH Ngb are crucial for its neuroprotective activity.

**Figure 7:** Protective effects of WT, H67V, E56Q, E63Q, and E121Q chimeric ZHHH Ngb proteins on PC12 cell death caused by hydrogen peroxide. WT, H67V, E56Q, E63Q, or E121Q chimeric ZHHH Ngb protein was applied to PC12 cells. Following treatment of the cells with hydrogen peroxide, cell viability was measured by MTS assays. All data are expressed as means ± SEM from four independent experiments, each performed in triplicate. Data were analyzed by one‐way ANOVA followed by Tukey–Kramer *post hoc* tests. **P < 0.01 compared with PBS. ^##^ *P* < 0.01 compared with WT chimeric ZHHH Ngb.

## Discussion

In this study, we demonstrated that chimeric ZHHH Ngb protein, in which the module M1 of human Ngb was replaced by that of zebrafish Ngb, has both cell membrane‐penetrating activity like zebrafish Ngb and neurite outgrowth‐inducing activity like human Ngb, suggesting that module M1 of zebrafish Ngb and modules M2‐M4 of human Ngb possess cell membrane‐penetrating and neurite outgrowth activities, respectively.

The neurite outgrowth‐inducing activity of chimeric ZHHH Ngb is similar to that of NGF, but their mechanisms differ from one another: NGF binds to its receptor, leading to the induction of neuronal differentiation and neurite outgrowth 33, whereas chimeric ZHHH Ngb binds to glycosaminoglycan and translocates into cells by macropinocytosis. Moreover, our previous studies demonstrated that chimeric ZHHH Ngb protects PC12 cells against oxidative stress‐induced cell death 10, 11, 12. Thus, chimeric ZHHH Ngb functions as a cell membrane‐penetrating inducer of neuroprotection and neuronal differentiation.

Recently, it was reported that overexpression of human Ngb promotes neurite outgrowth in mouse neuroblastoma N2a cells and in primary cultured rat cortical neurons 30 and that the overexpression of mouse Ngb in RGC‐5 cells significantly increases the length of neurite outgrowth 31. In addition, it was also noted that Ngb is expressed during neuronal differentiation of human embryonic stem cells *in vitro* and in the neurogenic subventricular zone of adult rats *in vivo* 37. Therefore, our results and these reports imply that mammalian Ngb plays crucial roles in neurogenesis as well as in neuroprotection under conditions of oxidative stress, such as ischemia and reperfusion.

In the present study, we investigated neurite outgrowth‐promoting activity under normoxia, during which most chimeric ZHHH Ngb forms a ferrous oxygen‐bound mono‐His conformation. During oxidative stress conditions, the ferrous oxygen‐bound mono‐His form of Ngb, which exists under normoxia, is converted to the ferric bis‐His conformation, inducing large tertiary structural changes. We previously clarified that ferric bis‐His Ngb, but not ferrous ligand‐bound Ngb, specifically binds to flotillin‐1, a lipid raft microdomain‐associated protein, as well as Gα_i/o_ 13, 16. Furthermore, by using a mutated Ngb protein that cannot form the bis‐His conformation, we demonstrated that the oxidative stress‐induced structural changes in human Ngb are essential for its neuroprotective activity. On the other hand, in the present study, we clarified that the neurite outgrowth‐inducing activity of chimeric ZHHH Ngb is not dependent on its heme environmental structural changes. These present results suggest that chimeric ZHHH Ngb or human Ngb interacts with molecules other than Gα_i/o_ or flotillin‐1 in the cells, leading to the induction of neurite outgrowth.

Glu53, Glu60, and Glu118 of human Ngb are crucial for its GDI and neuroprotective activities 10, 11, 13, 19, 21, 22. Sequence alignments among Ngb proteins from mammalia, aves, reptilia, amphibia, and osteichthyes showed that the Glu60 residue is conserved among all these species 22, Glu118 is conserved among mammalia, aves, reptilia, and amphibia 22, 28, and Glu53 is conserved only among boreoeutheria of mammalia, except for the harp or hooded seal 22, 28. The present results suggest that the Glu60 and Glu118, but not Glu53, residues of human Ngb are crucial for its neurite outgrowth‐inducing activity. Taken together, these results imply that the neurite outgrowth‐inducing activity of Ngb is evolutionally older than its neuroprotective activity.

## Author contributions

NT and KW conceived and designed experiments, analyzed data, and wrote the manuscript. NT, WO, and SW performed experiments.
